The article "Nanocarrier-Based Targeted Therapies for Myocardial Infarction" was published in 2022. Journal: Pharmaceutics.

# Nanocarrier-Based Targeted Therapies for Myocardial Infarction

**DOI:** 10.3390/pharmaceutics14050930

**Published:** 2022-04-25

**Authors:** Thomashire A. George, Chuan-Chih Hsu, Annette Meeson, David J. Lundy

**Affiliations:** 1 International Ph.D. Program in Biomedical Engineering, Taipei Medical University, Taipei 110, Taiwan; thomashireg@gmail.com; 2 Department of Cardiovascular Surgery, Taipei Medical University Hospital, Taipei 110, Taiwan; cchsu1967@tmu.edu.tw; 3 Biosciences Institute, Newcastle University, Newcastle upon Tyne NE1 3BZ, UK; annette.meeson@ncl.ac.uk; 4 Graduate Institute of Biomedical Materials and Tissue Engineering, Taipei Medical University, Taipei 110, Taiwan

**Keywords:** myocardial infarction, nanoparticle, liposome, exosome, ischemia

## Abstract

Myocardial infarction is a major cause of morbidity and mortality worldwide. Due to poor inherent regeneration of the adult mammalian myocardium and challenges with effective drug delivery, there has been little progress in regenerative therapies. Nanocarriers, including liposomes, nanoparticles, and exosomes, offer many potential advantages for the therapy of myocardial infarction, including improved delivery, retention, and prolonged activity of therapeutics. However, there are many challenges that have prevented the widespread clinical use of these technologies. This review aims to summarize significant principles and developments in the field, with a focus on nanocarriers using ligand-based or cell mimicry-based targeting. Lastly, a discussion of limitations and potential future direction is provided.

## 1. Introduction

### 1.1. Myocardial Infarction and Treatment Challenges

Ischemic heart disease is responsible for more deaths globally than all cancers combined [1]. Myocardial infarction (MI) is the single largest cause of death and has high mortality rates among both elderly and nonelderly (<65-year-old) adults [2,3]. Lifestyle and genetic factors result in atherosclerotic plaque buildup in the coronary arteries, which supply oxygenated blood to the myocardium [4,5]. These plaques can become unstable, resulting in sudden thrombus formation, which blocks blood flow and starves the myocardium of oxygen and respiratory substrates, resulting in cardiomyocyte (CM) necrosis and apoptosis [6]. In a typical adult human MI, up to a billion CMs are lost [7]. Adult mammals have exceptionally low rates of CM proliferation, resulting in poor regeneration following injury because parenchymal cells cannot be replaced in sufficient quantity [8]. Most acute MIs are not immediately fatal, but CMs are replaced by collagenous scar tissue, preserving the heart’s structural integrity but not contributing to contractile function. As a result of this cardiac remodeling, patients progress to heart failure [9]. 

The current gold-standard therapy following MI revolves around rapidly restoring blood flow using percutaneous coronary intervention (PCI) or thrombolytic drugs, followed by supportive treatments such as lipid-lowering agents and anti-hypertensives and anti-coagulants to reduce stress on the heart and reduce risk of future events [10]. A model treatment may revolve around the protection of CMs upon reperfusion and modulating long-term inflammation to reduce scar formation, promote angiogenesis and improve regeneration. However, there are no clinically used treatments that can directly stimulate cardiac regeneration [11].

### 1.2. Treatment Challenges

The complex MI pathogenesis, involving cell apoptosis, inflammation, and remodeling, has many steps which could potentially be exploited for therapeutic benefit. CM apoptosis may be reduced by agents such as insulin-like growth factor 1 (IGF-1), which activates the Akt pro-survival pathway [12]. Tissue perfusion may be improved by pro-angiogenic factors, such as vascular endothelial growth factor (VEGF), interleukin-8 (IL-8), and basic fibroblast growth factor (FGF-β), which can promote blood vessel formation, stabilization, and maturation [13,14]. Chemotactic molecules such as transforming growth factor (TGF)-β1, monocyte chemoattractant protein 1 (MCP-1), tumor necrosis factor-alpha (TNF-α), and granulocyte colony-stimulating factor (G-CSF) promote host monocyte recruitment and differentiation into macrophages, thus influencing local inflammation [15]. Tissue remodeling can be manipulated by altering the activity of matrix metalloprotease (MMP) and tissue inhibitors of metalloproteinases (TIMP) around the infarct area [16]. Anti-inflammatories, antioxidants, and immunomodulatory agents have also been explored as means to reduce damage following hypoxia and reperfusion [12]. There is also growing attention on the use of RNAs that play an important role in the normal physiology of the heart and are involved in angiogenesis, apoptosis, and fibrosis after myocardial infarction. Some RNAs may augment the resolution of the inflammatory progress, promoting cardiac repair [17]. However, these potential treatment modalities are hampered by poor delivery to the infarct area and the difficulty in achieving temporospatial control.

There are many reasons underlying poor myocardial delivery. Firstly, the heart itself is not easily accessible for drug administration. Myocardial uptake following intravenous administration is very low, which will be illustrated later in this review. Intramyocardial injection is the most direct route, but it requires invasive procedures and can carry higher risks due to the unstable nature of the ventricle wall after MI. Even then, therapeutics are rapidly lost into circulation, aided by vigorous contractions of the heart. This route is not amenable to a course of treatment that requires more than one injection since it is not practical to carry out multiple intramyocardial injections. 

A catheter can be used to deliver some types of therapeutics into the coronary artery, which supplies the myocardium. However, peptides such as VEGF or IGF-1 are rapidly degraded in the bloodstream or after direct injection into tissues [18,19]. Regeneration and remodeling occur over several months, with acute inflammation being both damaging and necessary for long-term wound healing. Therefore, it is unlikely that a single delivery of an isolated growth factor, cytokine, microRNA, or small molecules will be able to make a meaningful difference in long-term outcomes. In an ideal situation, the sustained delivery of multiple factors, in sync with the natural progression of inflammation and remodeling, would be required for true regeneration to occur. This is where advanced drug delivery technologies such as nanomedicines may offer useful contributions.

## 2. Nanomedicines and Nanocarriers

Nanomedicines are typically defined as materials with single diameters of less than 100 nanometers for diagnostic or therapeutic purposes [20]. This article focuses on the latter. Nanomedicines may function as stand-alone therapeutics if they can directly influence cell behavior or act as carriers for other therapeutics to improve their stability, delivery/targeting, or provide controlled release [21]. The repertoire of materials from which nanomedicines can be formulated is vast, including lipids (micelles, liposomes), metals (iron oxide, gold), polymers (polystyrene, poly (lactic-co-glycolic acid) (PLGA)), inorganics (silica) and proteins (albumin), to name a few [22]. Therapeutics can be encapsulated inside nanocarriers, or linked to their surface, and their release may be passive or triggered by certain stimuli, such as pH or enzyme activity. Nanomedicines targeting the heart can be administered by many routes, but intravenous, intracoronary, and intramyocardial delivery are commonly seen in the research literature. The scope of “nanomedicines” is beyond the scope of a single review article. Thus, this manuscript will focus specifically on nanocarriers rather than nanogels, nanofiber patches, nanotubes, and other technologies, which have been reviewed elsewhere [23].

Nanocarriers have many theoretical advantages for drug delivery, including the possibility of improved targeting and controlled/triggered release of therapeutics. For example, with appropriate formulation, liposomes can encapsulate substances that may have had poor pharmacokinetic properties alone. By modifying the liposome surface with compounds such as polyethylene glycol (PEG), the circulatory half-life can be extended, and accumulation of the drug (and subsequent toxicity) at undesired sites can be reduced. A well-known example is the chemotherapeutic Doxil^®^, the PEG-modified liposomal form of doxorubicin, which shows a greatly extended circulation time and an improved safety profile compared to the free drug [24].

A study by Chang and colleagues demonstrated that nanoparticles could reduce degradation and extend the biological activity of peptides in the myocardium [25]. PLGA nanoparticles of 60, 200 and 1000 nm were linked to IGF-1 by electrostatic forces to preserve IGF-1 structure and function. Following intramyocardial injection in a mouse MI model, the PLGA-IGF-1 nanoparticles retained IGF-1 at the infarct site and induced Akt phosphorylation (Akt-*p*) for up to 24 h. In comparison, free IGF-1 did not prolong Akt-*p* for longer than 8 h. As a result, the authors noted a small decrease in apoptotic CMs, increased cardiac function, and less scar formation due to the treatment.

Exosomes are nanoscale lipid membrane-bound extracellular vesicles secreted by cells and present in many body fluids, including blood, cerebrospinal fluid, urine, and breast milk [26]. Due to their natural origin, their membranes contain a wide variety of proteins, although they are typically identified by markers such as CD9, CD63, CD81, and recently syntenin-1 [27,28]. This membrane functionalizes exosomes with inherent targeting abilities due to their ability to interact with cells [29,30]. Exosome cargo is complex and, significantly, varies depending on the cell of origin. For example, as a generalization, stem cells from healthy donors may generally secrete pro-regenerative products, whereas diseased, injured, or cancerous cells may secrete products that reflect those conditions and negatively impact recipient cells [31,32]. Nevertheless, research has consistently shown that exosomes can function as potent therapeutics, cross biological barriers, interact with cells, and subsequently influence multiple biological pathways [31,33,34]. In addition, exosomes can be repurposed as drug delivery vehicles via loading with exogenous therapeutics or by engineering the parent cells to overexpress certain desired factors [29,35,36,37,38].

Nanomedicine utilizes two main strategies to target diseased organs or tissue. Passive targeting is based on physicochemical properties and the enhanced permeability and retention (EPR) effect, or active targeting, which uses ligands such as peptides, antibodies, polysaccharides, proteins, aptamers, and small molecules [22]. Nanocarriers can be designed to display these targeting moieties, allowing them to bind to specific targets, thus increasing their retention at the delivery site. There has also been increasing interest in nanocarriers bearing magnetic bio-probes for enhanced targeting in the past decade, which are reviewed elsewhere [39].

## 3. Nanomedicines for Cardiac Therapy

### 3.1. Passive Targeting

In terms of drug delivery, many nanocarriers rely on the EPR effect to reach the desired target site via extravasation from the blood. The EPR effect occurs due to abnormal or highly permeable vasculature at sites of injury or inflammation. In the case of solid tumors, where the EPR effect was first described, the rapid proliferation of cancer cells increases oxygen demand and requires vascularization; thus, chaotic, leaky vessels are laid down [40]. However, the EPR effect following MI does not evolve by the same mechanism. During MI, there is a rapid loss of cardiac cells, including cardiac endothelial cells. The release of cytokines increases local vascular permeability and inflammation, resulting in an EPR effect. This is used experimentally to measure the “area at risk” by detecting the extravasation of dyes or contrast agents, thus showing the affected region [41]. Several preclinical studies have reported success with passive targeting of the cardiac myocardium post-infarction, improving cardiac functions [42,43,44,45]. However, the infarcted myocardium has a relatively poor EPR effect for nanomedicines, as shown in Figure 1. A study by our group investigated the biodistribution of fluorescent-labeled PEG-modified nanoparticles (20, 100, 200, 500, 1000, and 2000 nm) following ischemia-reperfusion (I/R) injury in mice [46]. Nanoparticles were allowed to circulate for 30 min; then, the mouse vascular network was perfused to remove unbound nanoparticles from the vessels, and tissues were sampled. The fluorescent dye was quantified by a validated high-performance liquid chromatography (HPLC) method, providing sensitive measurements of nanoparticle uptake. In the healthy myocardium, only 0.029% of injected 20 nm nanoparticles were retained. Following I/R injury, this increased by approximately 5.5-fold, showing that an EPR effect is indeed present in the infarcted left ventricle. Though this increase was statistically significant, it represents such a low level of nanomedicine delivery (less than 0.2%) that it is unlikely to be clinically meaningful. For context, the spleen and liver together retained more than 50% of the injected nanoparticles. The greatest total uptake by the heart after MI (0.27%) was found using 500 nm nanoparticles; however, confocal microscopy revealed that most of these nanoparticles were lodged inside small capillaries rather than in the myocardium itself. 

We concluded that nanoparticles of approximately 100 nm offered the best overall uptake and delivery to the target area, but passive uptake following intravenous injection was very low in our model system. In addition, previous studies have demonstrated that the EPR effect following ischemic injury may be short-lived and vessel permeability is normalized within a few days [47,48]. As mentioned earlier, in the context of inflammation and remodeling, which resolves over several months, the EPR effect does not offer a long-term solution for MI therapy. Therefore, there is a strong rationale for designing targeted nanomedicines that can improve delivery beyond passive uptake.

### 3.2. Active Targeting

Nanocarriers can be designed to actively target specific tissues or cells, sparing normal tissues and limiting side effects. Ligand-based targeting seeks to exploit targets that are highly enriched in the target site compared to the rest of the body. For the infarcted heart, this may include CM surface receptors or structural proteins or markers of inflammation and cell damage that are elevated in the local area following injury. Several targeted nanocarriers have been designed, and in vivo and in vitro preclinical studies have reported increased delivery, retention and efficacy in the ischemic heart compared to nontargeted carriers. This review aims to highlight studies that demonstrated targeted nanocarriers used for treatment of myocardial infarction. Each will be discussed based on the material used to fabricate the carriers. A summary of 20 key studies is shown in Table 1.

#### 3.2.1. Polymer-Based Nanocarriers

Polymeric nanocarriers have high stability, bioavailability, and innate potential for sustained drug release kinetics [49]. They are also versatile, and can accommodate a wide range of molecules. Polymeric nanocarriers can protect the encapsulated drug and offer a controlled and sustained drug release profile. This has been attributed to the fact that the rate of polymer biodegradation and diffusion of the drug from the polymer matrix can be regulated [49]. As described above, a sustained release of active therapeutic is needed to ensure maximum protection of cardiac cells and regeneration, and to achieve improvements in heart function.

PLGA is an approved material by the Food and Drug Administration (FDA) and the European Medicines Agency (EMA) for the engineering of pharmaceutical products, being highly biodegradable and biocompatible [50]. It has been shown to have a high affinity for inflammatory tissues targeting inflammatory monocytes, thus promoting its capacity to target cardiomyocytes after MI because there is increased migration of inflammatory cells and monocytes to the heart post-infarction [51]. Nakano and colleagues showed that intravenously injected PLGA-nanoparticles accumulated in the infarct region following an ischemia/reperfusion injury (IR), but were not distributed to the normal heart [52]. In this study, irbesartan-loaded PLGA-based nanoparticles showed a threefold increase in irbesartan concentrations in the ischemic myocardium compared to normal myocardium in IR mice model, and a 17-fold increase compared to the free drug.

Surfaces of nanocarriers are often coated with polyethylene glycol (PEG) to reduce opsonization, increase circulation time and increase accumulation at the target site. Currently, active targeting is combined with formulations enhancing passive targeting. In a recent study, Sun et al. reported that an arginine–glycine–aspartic acid tripeptide (RGD)-modified polyethylene glycol (PEG)-polylactic acid (PLA) nanocarrier was effective in delivering miR-133 to the infarcted heart, sparing normal tissues [53]. Studies have shown that RGD tripeptide can bind to activated platelets, making it suitable for the targeting of post-infarcted cardiac tissue, as it has been established that platelet activation is a key player in cardiac damage that follows an ischemic attack [54].

Zhang and colleagues designed a nanocarrier combining Szeto-Schiller 31 (SS31), a mitochondria-targeting peptide, with PLGA and PEG [67]. SS31 is a synthetic peptide that binds specifically to cardiolipin (CL) within mitochondria. This enables targeting since there is mitochondrial damage following an ischemic attack with disruption of ATP production, leading to the opening of the mitochondrial permeability transition pore. This nanocarrier, CsA@PLGA-PEG-SS31, was shown to increase the delivery of Cyclosporin A (CsA) to cardiomyocytes after IV injection in a rat I/R model. This treatment reduced infarct size by approximately 50% and reduced apoptosis compared to free CsA administration, exhibiting cardioprotective effects in myocardial reperfusion rats, decreased apoptosis and reduced cardiac remodeling. Intravenous lipid-encapsulated CsA was previously explored in a human clinical trial but failed to improve outcomes following MI [69].

Xue et al. reported a myocardium-targeting PEGylated dendrigraft poly-L-lysine (DGL) with angiotensin II type 1 (AT1) to form AT1-PEG-DGL, a ~200 nm nanovector [57]. Angiotensin II type-1 receptors (AT1R) are highly expressed soon after MI, making them suitable targets for nanocarrier delivery. The authors showed that AT1-PEG-DGL quickly accumulated in the ischemic heart 30 min following IV administration, peaked at one-hour post-injection, and showed longer retention compared to the non-targeted dendrimer. AT1-PEG-DGL was used to carry an microRNA-1 antisense oligonucleotide (AMO-1) to the heart following MI surgery in mice, resulting in reduced CM apoptosis and infarct size. Dendrimers have also been shown to be suitable candidates for gene delivery, owing to their highly branched structure and enhanced flexibility [70].

Díaz-Herráez et al. designed a system that combined polymeric microparticles (MPs) loaded with neuregulin (NRG) adhered to adipose-derived stem cells (ADSCs) [71]. This ADSC-NRG-MP treatment was shown to prolong cell survival in the heart for up to 3 months and improved therapeutic outcomes in a rat MI model, offering a major advantage in MI therapy.

The release kinetics of a nanocarrier can also be controlled by including stimuli-responsive elements to release drugs upon exposure to biological factors such as pH changes or enzyme activity. Karen Christman’s group developed polymeric enzyme-responsive nanoparticles which aggregate into a scaffold upon exposure to MMP-2/9. Although these nanoparticles still rely on the EPR effect, enzyme-responsivity substantially increased their retention in the infarct area following intravenous administration in a rat MI model. Nanoparticle aggregates were still retained in the infarct area 28 days following administration, whereas non-enzyme-responsive particles were rapidly cleared within hours [55].

Polymeric micelles have also proven to be effective nanocarriers for administration via different routes due to their small size, good solubility, and ease of preparation [72]. However, there are still unmet challenges. Although they are mostly biodegradable, there are potential toxicities associated with some of their components. There is also the need for a better understanding of their physicochemical behavior [73]. In addition, despite most papers reporting improved drug delivery compared to free drugs, the percentage is still typically less than 3–5%.

#### 3.2.2. Lipid-Based Nanocarriers

Lipid-based nanocarriers are biocompatible, have high bioavailability, and can carry both hydrophilic and hydrophobic compounds. They have a wide range of physicochemical properties that can be tuned to regulate their biological characteristics. These properties, coupled with the relative simplicity of its formulation, scale-up, and low production cost, make them very useful in target-specific therapy [74]. Lipid nanocarriers have been extensively studied and are clinically used in applications such as cancer. They are also promising candidates for drug delivery to the infarcted heart [22,75]. Their circulatory properties can also be modified by conjugating the surface with PEG, which helps to prevent phagocytic clearance and prolong circulation time, thus increasing their capacity for passive targeting. Other factors that affect passive targeting are the size, polarity of lipid head group, membrane rigidity, and mechanical properties [44,76]. Lipid-based nanocarriers have been shown to successfully deliver cardioprotective drugs to the infarcted myocardium by passive targeting after IV administration [45]. Nevertheless, researchers have investigated the functionalization of lipid nanocarriers with affinity ligands such as peptides and antibodies to promote active targeting.

Primary Cardiomyocyte peptide (PCM) is a 20 amino acid (WLSEAGPVVTVRALRGTGSW) peptide being explored for ligand-based targeting in MI therapy. PCM was identified by phage display as having highly selective targeting of primary cardiomyocytes. However, it has low cell penetration as it interacts with an extracellular matrix protein tenascin-X [77]. Wang X. et al. designed a dual-ligand-modified liposomal nanocarrier (approximately 110 nm) using PCM in combination with a cell-penetrating peptide (transactivating transcriptional activator (TAT)), thus improving the internalization efficiency [78]. Synergistic interaction was demonstrated between both peptides. The dual-labeled liposomes showed a two-fold increase in targeting efficiency, measured by flow cytometry, compared to the unlabeled or single-labeled liposomes in vitro neonatal cardiomyocytes. Similar improvements were noted in a mouse model following IV administration. However, the authors did not use a myocardial infarction injury model, and so the results show uptake without the influence of injury-induced EPR effects.

Lipid nanoparticles (LNPs) are another subset of lipid-based nanocarriers. These gained increased recognition after the approval of Onpattro, the first RNAi-based therapeutics for clinical use. These form micellar structures and are effective for delivering nucleic acids [74]. Yu and colleagues designed an adenosine-loaded lipid nanocarrier with a lipid core and hydrophilic shell, which enables atrial natriuretic peptide (ANP), the targeting ligand, to be attached to the surface [68]. ANP is a member of the natriuretic peptic family that binds specifically to natriuretic peptide receptors (NPRs) that are over-expressed in the endocardium of the ischemic heart. The ANP-modified lipid carriers displayed significantly greater uptake and retention by rat cardiac (H9C2) cells, and moderately higher (approximately 1.5-fold) uptake by the infarcted heart, compared to the unlabeled carrier, showing a slight benefit over EPR-based delivery.

There is increasing research interest in dual ligand targeting, with some systems being designed for targeting different cells or cell compartments and some dual-ligand modified nanocarriers designed to target different receptors on the surface of the same cell. The latter has the advantage of achieving a synergistic effect by improving specificity and uptake. Wang and colleagues designed a dual ligand modified co-loaded lipid polymer hybrid nanoparticle (LPN) functionalizing with triphenylphosphonium (TPP) and ANP. TPP, being cationic, can accumulate several hundred-fold within the mitochondrial, passing readily through its high negative membrane potential. The dual-modified LPN, termed ANP/TPP-BN-LPNs, was loaded with baicalin, which has anti-apoptotic properties. Using a rat MI model, the authors targeted nanoparticles showed an approximate 5.5-fold increased delivery of the drug compared to the free molecule. The addition of dual-targeting improved delivery approximately threefold compared to non-targeted nanoparticles [79].

Lipid polymer hybrid nanoparticles (LPN) are a core–shell drug delivery system that combines the properties of polymeric and liposomal nanoparticles. This system enables the functionalization of hydrophilic shells with the benefit of a lipid core for insoluble drugs. They have been shown to enhance physical stability and increase loading capacity with greater control over drug release; surface functionalization is easier, and they can be converted to smart delivery vehicles [80].

Antibodies have a high affinity for a specific antigen and can be conjugated to many types of nanocarrier, enhancing their targeting specificity [81]. Antibody-modified liposomes have been reported to be effective in targeting myocardial infarction [59]. Cardiac troponins are highly expressed in cardiomyocyte cytoplasm, are released upon cardiac damage, and are used as a standard marker for the diagnosis of MI [82]. Li and colleagues developed a PEGylated liposome nanocarrier conjugated with antibodies against cardiac troponin T (cTnT) to deliver microRNA-21 mimics to the infarcted heart [63]. MicroRNAs (miRNA) are small, non-coding RNAs that are known to interact with several protein-coding genes, mediating a diverse spectrum of normal and pathological processes involving the heart. This pleiotropic ability has led to them emerging as suitable candidates for MI therapy [83]. However, free miRNAs are very unstable in circulation and have poor cellular uptake—hence the rationale for delivery via nanocarrier. The study showed that encapsulated miR-21 mimics induced a 2.15-fold higher expression of myocardial miR-21 compared to free miR-21 mimics or saline-administered controls. This was further increased to 3.48-fold upon the addition of CtnT-targeting antibodies, resulting in a higher ejection fraction and reduced infarct size.

Antibodies against chemokine receptors have also proven suitable for targeting the infarcted myocardium. Wang et al. loaded lipid micelles with a CCR2 antagonist and then functionalized them with an anti-CCR2 antibody [58]. The labeled micelles showed increased accumulation compared to the unlabeled micelles, and the CCR2 antagonist reduced inflammatory macrophage recruitment and infarct size in a mouse MI model.

Aptamers are synthetic, short, single-stranded DNA or RNA molecules that can selectively bind to specific cells or targets [84]. As described earlier, dynamic recruitment of neutrophils, monocytes, and macrophages to the infarcted site occur following myocardial infarction. Patrick Hsieh’s group designed a system for targeting recruited monocytes using lipid nanoparticles that could selectively bind to the surface of the circulating monocytes, which deliver the nanocarrier to the infarcted site [66]. In this study, aptamers were selected for strong binding to two macrophage cell lines and selected for weak binding to endothelial cells to avoid interaction with blood vessels following administration. Aptamers were then attached to DSPE-based lipid nanoparticles containing IOX2. IOX2 is a selective hypoxia-inducible factor 1 alpha (HIF-1a) prolyl hydroxylase-2 inhibitor, protecting HIF-1a from degradation and thus reducing CM apoptosis. Using this strategy, approximately 5% of the injected nanoparticles reached the infarct site, which is much higher than could be achieved by EPR-based uptake alone.

Other studies have utilized similar strategies where host cells are used to deliver nanocarriers to the infarcted heart, which will be discussed later in the paper. Ben-Mordechai and colleagues showed that hyaluronan-modified lipid nanoparticles have a high affinity for macrophages and can promote the targeting of infarcted hearts for MI therapy. Nanoparticles, loaded with heme oxygenase (HO-1) activator hemin, polarized infarct macrophages towards the anti-inflammatory “M2” phenotype, reduced infarct size, increased angiogenesis and improved echocardiography parameters [65].

#### 3.2.3. Inorganic Nanocarriers

Inorganic carriers can be precisely formulated with a wide range of sizes, structures, and geometry and have been found to be relatively more stable than other nanocarriers. They are characterized by a large surface area and can be modified with facile preparation [74]. They are made from inorganic materials, including gold, iron, or silica, with unique physical, magnetic and electrical properties acquired from the parent material. One inorganic nanoparticle that has shown great promise in targeted therapy are mesoporous silica nanoparticles (MSNs). MSNs have several advantages, including relative simplicity of functionalization, high stability and a large surface area and pore volume to load therapeutics [85]. Ferreira and colleagues fabricated a PEGylated porous silicon (Psi) nanocarrier (approximately 200 nm) functionalized with atrial natriuretic peptide (ANP) for delivery of cardioprotective drugs to the infarcted myocardium [56]. ANP can bind specifically to receptors overexpressed in the ischemic endocardium and can also reduce the extent of IR injury and subsequent infarct size [80]. Psi was biocompatible and biodegradable, and PEGylation markedly enhanced their stability. Primary rat neonatal cardiomyocytes and non-myocytes, pretreated with cobalt chloride to mimic a hypoxic state, retained 50–70% more ANP labeled Psi than the unlabeled Psi in in vitro studies. Single-photon emission computed tomography (SPECT/CT) imaging and autoradiography showed that, compared to unlabeled nanocarriers, the Psi-ANP nanocarrier was highly retained in the endocardial layer of the left ventricle of ischemic rat models within 10 min of intravenous administration. To demonstrate therapeutic utility, the authors loaded the nanoparticles with a small molecule, trisubstituted-3,4,5-isoxazole (C1), which was able to decrease ERK1/2 phosphorylation in an isoproterenol-induced ischemia model.

### 3.3. Cell-Based and Biomimicry-Based Targeting

Following MI and cell death, pro-inflammatory cytokines are released, attracting circulating immune cells to the damaged area. Neutrophils are recruited by a process dependent on chemokine (C-X-C motif) ligand 1 (CXCL1) and CXCL8 within the first hours after MI, and peak after approximately 24 h [86]. Monocytes from circulation are recruited to the heart, as are splenic monocytes, which are a major contributor of macrophages in the infarcted heart. Upon arrival, monocytes differentiate into macrophages which play multiple roles such as removing dead cell debris, but also participating in pathogenic remodeling. Monocyte recruitment to the heart peaks at approximately 72 h and lasts for approximately two weeks. The recruitment occurs in a biphasic manner, with earlier cells partaking in inflammation and digestion of damaged tissue; later, the cells play an anti-inflammatory role (secreting VEGF, interleukin-10, and others) [87]. These processes may be exploited by targeting nanomedicines against macrophages or other recruited cells, thus using them as a convenient, targeted delivery vehicle to deliver therapeutics to the infarct area.

Bejerano et al., exploring this premise, designed a miRNA-21-carrying nanoparticle conjugated with Ca^2+^ and hyaluronan-sulfate (HAS) to target post-MI macrophages [17]. The HAS-Ca^2+^-miRNA nanoparticle was found to be stable; it effectively targeted post-MI macrophages and significantly increased the expression of anti-inflammatory genes compared to non-targeted nanoparticles.

Evidence has shown the mobilization of CD34^+^-expressing cells following acute myocardial ischemia with subsequent engraftment and retention in the ischemic myocardium [88]. Although this paper attracted some criticism, these cells appeared to promote angiogenesis through paracrine secretions and mediate the repair of ischemic tissue. A later study by another group showed that CD34^+^ cell-secreted membrane-bound nano-vesicles (CD34Exo) were also shown to target ischemic tissues [89]. Activation of platelets following MI leads to the formation of platelet/CD34^+^ cell coaggregates, enhancing chemotaxis, adhesion, and MI-homing capacity [90].

Platelets (thrombocytes) are also known to interact with circulating monocytes, and so platelet membrane extracts, rich in monocyte-interacting proteins (GPIIb, CD36, CD42b, JAM-C, etc.), have been linked to liposomes as a targeting mechanism. Using platelet-like proteoliposomes in a mouse model of I/R, Cheng and colleagues observed a roughly 17-fold increase in delivery (approximately 5% of total injected liposomes) compared to liposomes without platelet protein membranes [91]. Using naturally derived membranes as a targeting mechanism is advantageous in many ways since the combination of multiple ligands is able to better recapitulate the natural biology and can provide more specific binding to desired targets.

The inherent ability of platelets to target ischemic injuries was evaluated by Tang et al. They showed increased retention of platelets in the MI heart compared to the sham after intravenous injection [92]. In this study, platelet nanovesicles (PNV) displaying distinct platelet surface markers (CD42b (GPIbα), GPVI, and CD36 (GPIV)) were fused onto the membranes of cardiac stem cells (CSCs) to form PNV-CSCs. There was enhanced targeting and retention in the rat model of ischemia/reperfusion injury, which translated into increased therapeutic efficacy of CSCs. These effects were further confirmed in a porcine model of ischemia/reperfusion.

These strategies are highly promising, and targeting based on exploiting host cell recruitment appears to provide greater nanocarrier delivery to the myocardium and does not rely on the EPR effect. However, relying on natural cell membranes or membrane extracts to provide targeting has inherent limitations. A platelet or cell possesses hundreds of proteins on its surface, which are also often modified by glycosylation [93]. Isolation, purification, storage, and nanocarrier-coating methods may cause variation between batches, and standardizing a final pharmaceutical product is challenging.

A summary of EPR-dependent and targeting-based strategies is presented in Figure 2.

### 3.4. Exosomes for Cardiac Therapy

Exosomes offer many theoretical advantages for the therapy of myocardial infarction. As described earlier, exosomes function as naturally derived nanocarriers containing complex payloads that reflect the properties of the originating cell. Since the benefits of cell therapy appear to be driven primarily by paracrine effects, exosomes may provide many of the benefits of cell therapy, without the requirement to isolate, purify, culture, store and administer live cells [94,95]. Exosome-based therapy also has fewer concerns over immune rejection and tumorigenesis than stem cell therapy. Finally, their small size and cell-derived membranes allow them to be safely administered by intravenous injection with some targeting capability. Exosomes from many sources have been explored for cardiac therapy, including bone marrow, adipose, and umbilical-derived mesenchymal stromal cells (MSCs) [96]. In addition, exosomes from cardiosphere-derived cells (CDC) and iPSC-derived cardiomyocytes have been examined.

Vandergriff and colleagues conjugated cardiosphere-derived stem cells (CDCs) with cardiac homing peptide (CHP) [97]. There is evidence that CDCs can induce myocardial regeneration by transporting miRNAs to the myocardium. Cardiac-homing peptide (CHP) with the sequence CSTSMLKAC was identified by phage display as having high selectivity for the ischemic myocardium [98]. The authors in this study showed significantly increased uptake of modified exosomes (CHP-XO) compared to control exosomes conjugated with scrambled non-specific peptides. Echocardiography showed that treatment with CHP-XO resulted in improved heart function and reduced infarct area in a rat IR model.

Similarly, Wang and colleagues demonstrated that exosomes could be modified with the same peptide (CSTSMLKAC), which they termed ischemic myocardium-targeting peptide (IMTP) [99]. Exosomes derived from cultured mouse mesenchymal stem cells modified to overexpress IMTP displayed an improved uptake in H9C2 (rat cardiomyoblast) cells in vitro and in a C57BL/6 mouse model. Exosomes were administered by intravenous injection and showed an approximately twofold increase in the infarct area compared to unmodified exosomes, which shows that some targeting beyond the EPR effect was achieved. This was accompanied by decreased local inflammation, increased angiogenesis, and reduced apoptosis. In this instance, mice administered PBS only displayed approximately 28% of apoptotic myocardial cells, unlabeled exosomes approximately 11%, and targeted exosomes approximately 5%.

An important study by Eduardo Marban’s group [100] examined human cardiosphere-derived cell exosomes in a pig MI model administered at short (30 min) and long (four weeks) time points after injury. CDCs have been previously shown to have numerous benefits in animal studies and human clinical trials, such as reduced scar formation and improved myocardial preservation [101]. CDC-derived exosomes have also been shown to contain beneficial RNAs, which have potential benefits in in vitro assays [102,103]. Therefore, it was hypothesized that CDC-derived exosomes may provide similar benefits in a clinically relevant MI model. This study demonstrated that intracoronary exosomes provided much more variable results and no overall statistically significant benefits. However, direct intramyocardial injection significantly reduced infarct size and increased ejection fraction % in a consistent manner. This was directly related to delivery efficiency, with labeled exosomes showing less retention at the injury site following intracoronary injection. This clearly illustrates the importance of drug delivery for nanocarrier-based therapies, whereupon effective treatments fail due to poor retention at the target site.

Exosome therapy is not without its limitations, however. Exosome origin is critical. A recent study demonstrated that exosomes derived from heart failure patient tissues contained miRNAs, which had negative effects on pro-angiogenic and anti-apoptotic functions [104]. Another recent study showed that extracellular vesicles derived from post-MI hearts modulated macrophages towards the M1 phenotype and worsened cardiac injury in animal MI models [32]. Thus, it is clear that there are optimal and suboptimal donors which produce very different final “products”. In addition, the isolation, purification, and storage methods vary by throughput and cost, and produce exosomes of varying purity, as do standards for characterizing concentrations and administration dose [105,106]. These issues are reviewed in greater detail elsewhere [35,36,107].

## 4. Limitations and Future Challenges

The inherent low regeneration of the adult mammalian myocardium, the complex disease pathogenesis, and poor drug delivery and retention are all significant obstacles to effective therapies. It is notable that across the papers reviewed, nanocarrier encapsulation itself is often beneficial, improving therapeutic delivery and efficacy beyond the free substance. The addition of ligand-based targeting typically provides additional improvements in drug delivery in the range of two- to fivefold in animal models. Strategies using host cell-based delivery have shown greater increases in an EPR-independent manner. The cited studies using peptides, miRNAs, and small molecules have shown reductions in infarct size, reduced scarring, increased angiogenesis, and improved echocardiography parameters in mouse or rat MI models. Thus, there is no shortage of interventions that may be potentially useful. 

However, experimental animal models have some limitations. Many experiments are carried out using left anterior descending (LAD) coronary artery ligation in young C57/BL6 mice or Wistar rats. This contrasts with MI patients, who are typically older and possess multiple co-morbidities that affect their outcome. Studies have shown that older animals have different cellular responses following MI surgery, including increased CM apoptosis and subsequent reduced effectiveness of caspase inhibition (anti-apoptotic) therapies [108,109]. Many other variables have been identified, including mouse strain, anesthesia methods, artery ligation method, and even the time of day at which the surgery is performed [110].

In terms of drug delivery, mouse tissues are much smaller in volume, and a typical LAD ligation creates an infarct covering 35–60% of the entire left ventricle [111]. Furthermore, the entire murine left ventricle can be easily covered with 3–4 intramyocardial injections. In larger animal models such as mini pigs (approximately 25 kg), more than 20 intramyocardial injections are needed to cover the infarct and border zone [112]. This can be performed by percutaneous intramyocardial injection, or via a second thoracotomy procedure. There are some risks associated with intramyocardial injection, particularly during the period when the ventricular wall is unstable following injury. Mice also have a small blood volume and rapid circulation compared to large animals or human patients, which enables greater delivery and uptake of bloodborne nanomedicines. Injury location, onset, and the timescale of disease progression are also different between mice and large animals or humans [113]. In mice, LAD ligation affects the free wall primarily, whereas, in minipigs, the intraventricular septum is affected. These differences result in altered findings by echocardiography and intraventricular catheterization. A thorough overview of model cardiovascular systems is provided elsewhere [114]. 

Lastly, for nanocarriers there must be clear standardization of the materials, characterization methods, administration routes and regulatory recognition [20]. This is complicated further in the case of biological products such as exosomes. One-fifth of US FDA-approved nanodrugs are indicated for cancer therapy, and there are no approved nanodrugs for the treatment of MI. Two nanoparticles are approved for post-MI imaging application [115,116], and a clinical trial to investigate liposomal methotrexate (NCT03516903) following MI was recently terminated due to the COVID-19 pandemic.

## 5. Conclusions

Due to poor endogenous regeneration of the adult mammalian heart after injury, new treatments for myocardial infarction are urgently needed. Such treatments may aim to reduce cardiac cell loss, modulate remodeling, or promote regeneration. Many growth factors, cytokines, and small molecules have demonstrated these capabilities; however, they are limited by poor delivery, uptake, and retention at the target site, and the myocardial EPR effect is relatively mild and short-lived. Thus, nanocarriers offer a potential solution, particularly if they can use active and EPR-independent means of targeting the injured area. Many strategies are being actively researched, including ligand-based targeting, biomimicry to exploit immune cell recruitment, and the use of exosomes as naturally targeted delivery vehicles. However, there are many more obstacles to cross before these technologies can be translated to widespread clinical use.

## Figures and Tables

**Figure 1:** Passive EPR-based nanoparticle retention by the infarcted heart is low. The coronary artery was occluded for 45 min, then the blood flow was restored to create an ischemia-reperfusion injury. Thirty minutes after myocardial reperfusion, PEG-modified polystyrene nanoparticles bearing a green fluorescent dye were administered by the tail vein. Uptake was quantified by HPLC and fluorescence microscopy. The results showed that nanoparticle uptake by the infarcted heart was greater than sham but represented less than 1% of the injected nanoparticle dose. ns = not significant, ** = *p* ≤ 0.01, **** = *p* ≤ 0.0001. Figure reproduced from [46].

**Figure 2:** A summary of selected promising nanocarrier drug delivery strategies is shown. Nanocarriers carry payloads of single or multiple small molecules, miRNAs, or peptides with diverse effects. Some examples of targeting strategies are shown. Modification of the nanocarrier can be accomplished by the use of specific antibodies, targeting peptides (PCM—primary cardiomyocyte; IMTP—ischemic myocardial targeting peptide) or aptamers. Targets include AT1, NPR, or troponin, which are increased following MI. Biomimicry techniques such as membrane cloaking enable EPR-independent delivery via circulating immune cells.

**Table 1:** Summary of nanocarriers utilized for myocardial infarction therapy.

Targeting	Nanocarrier/Payload	Findings	Ref.
Passive/EPR Intravenous	PLGA NPs/irbesartan	Reduced infarct size vs. free drug (mouse)	[52]
Passive/EPR Direct injection	PLGA NPs/VEGF	Improved cardiac performance and vascular density (mouse)	[21]
Passive/EPR Intravenous	Copolymer micelles/TEMPO ^1^	Reduced infarct size, apoptosis, (canine I/R model)	[43]
Passive/EPR	Liposome/berberine	Preserved cardiac function (mouse) compared to free Berberine	[44]
Passive/EPR	Liposome/tanshinone and puerarin	Improved drug delivery to heart compared to free drug (rat)	[42]
Passive/EPR	Liposome/modRNA	Delivery and expression of functional protein at infarct site following intravenous injection(mouse)	[45]
Responsive/EPR	MMP-responsive NPs	Improved retention in infarcted myocardium (rat)	[55]
Ligand-based (ANP)	Porous silica NPs	Improved retention in ischemic left ventricle (rat)	[56]
Ligand-based (AT1)	Dendrimer/AMO ^2^	Improved delivery vs. non-targeted. Reduced apoptosis and infarct size (mouse)	[57]
Ligand-based (anti-CCR2 antibody)	PEG-DSPE micelle/ CCR2 antagonist	Reduced inflammatory cell recruitment and infarct size	[58]
Ligand-based (anti-Troponin antibody)	Liposome/AMO ^2^	Increased delivery to infarct area compared to non-targeted liposomes (rat)	[59]
Ligand-based (RGD)	Liposome/Peurarin	Increased delivery to heart, reduced infarct size (rat)	[60]
Ligand-based (multiple targeting peptides)	Liposome/ PARP inhibitor	Ninefold higher delivery to cardiomyocytes than non-targeted peptides (mouse)	[61]
Ligand-based (MMP targeting peptide)	Micelle/ MMP-targeting peptide	Increased micelle delivery to infarct area compared to non-targeted micelles (mouse)	[62]
Ligand-based (anti-troponin antibody)	Liposome/miR-21	Increased binding and retention in heart (rat)	[63]
Ligand-based (MMP-targeting peptide)	Lipid NPs/ schisandrin B	Slightly improved drug delivery and reduced infarct size (rat)	[64]
Cell/Ligand-based (hyaluronan)	Liposome/hemin	Targeting macrophages to deliver to infarcted heart. Improved cardiac function, angiogenesis and reduced scar vs. free drug (mouse)	[65]
Ligand-based (RGD)	PEG + PLA NPs/ miR-133	Slightly improved vs. free miRNA or non-targeted liposomes (mouse)	[53]
Ligand-based (aptamer)	Liposome/IOX2	Delivered to ischemic heart via macrophages. Improved cardiac function (mouse)	[66]
Ligand-based (mitochondria-targeting peptide)	PLGA/cyclosporine A	Passive targeting combined with active targeting of the mitochondria. Increased accumulation in ischemia compared to normal (rat)	[67]
Ligand-based (ANP)	Lipid NP/adenosine	Improved delivery and reduced infarct size (rat)	[68]

^1^ 2,2,6,6-tetramethylpiperidine-1-oxyl. ^2^ anti-miR-1 antisense oligonucleotide.
